The article "A Neuron-Glial Model of Exosomal Release in the Onset and Progression of Alzheimer's Disease" was published in 2021. Journal: Front Comput Neurosci.

# A Neuron-Glial Model of Exosomal Release in the Onset and Progression of Alzheimer's Disease

**DOI:** 10.3389/fncom.2021.653097

**Published:** 2021-09-20

**Authors:** Hina Shaheen, Sundeep Singh, Roderick Melnik

**Affiliations:** ^1^M3AI Laboratory, MS2Discovery Interdisciplinary Research Institute, Wilfrid Laurier University, Waterloo, ON, Canada; ^2^BCAM-Basque Center for Applied Mathematics, Bilbao, Spain

**Keywords:** brain, calcium channels, exosomes and biomarkers, molecular communication, temperature effects, astrocytes, dynamic models, Alzheimer's disease

## Abstract

Exosomes are nano-sized extracellular vesicles that perform a variety of biological functions linked to the pathogenesis of various neurodegenerative disorders. In Alzheimer's disease (AD), for examples, exosomes are responsible for the release of *Aβ* oligomers, and their extracellular accumulation, although the underpinning molecular machinery remains elusive. We propose a novel model for Alzheimer's *Aβ* accumulation based on *Ca*^2+^-dependent exosome release from astrocytes. Moreover, we exploit our model to assess how temperature dependence of exosome release could interact with *Aβ* neurotoxicity. We predict that voltage-gated *Ca*^2+^ channels (VGCCs) along with the transient-receptor potential M8 (TRPM8) channel are crucial molecular components in Alzheimer's progression.

## 1. Introduction

Protein misfolding, oligomerization, and aggregation are responsible for the initiation of pathological disorders in the brain (Soto and Pritzkow, 2018). Nano-sized extracellular vesicles (exosomes) are believed to be key mediators in the transfer of cytotoxic proteins between the nerve cells, resulting in the spread of many neurodegenerative diseases, such as Alzheimer's disease (AD), Parkinson's disease (PD), Huntington's disease (HD), and Creutzfeldt-Jacob's disease (CJD) (Jiang et al., 2019; Luo et al., 2020; Zhang and Wang, 2020).

Exosome releases increased intracellular calcium (*Ca*^2+^) (Jain, 2019). Specifically, Veletić et al. (2019) have shown that depolarization of neurons and glial cells, such as astrocytes, can trigger multivesicular exosome release therefrom. Because neurons interact with astrocytes and vice versa through a plethora of ion and molecular pathways that can reciprocally affect their membrane electrical potential (De Pittà, 2020), a question arises whether this interaction could be physiologically relevant for exosome release in the brain.

In AD etiology, oligomeric *Aβ* can substantially affect intracellular *Ca*^2+^ homeostasis both in neurons and in astrocytes (Bezprozvanny and Mattson, 2008; Shigetomi et al., 2016), thereby potentially regulating exosome release too. The mechanism whereby this could happen and the relevant pathogenic factors are not known. The reason for this gap of knowledge is because of inherent limits in the available technology, and because the biophysical framework to account for exosomal release in the neuropil in the context of neuron-glial interactions is missing (De Pittà and Berry, 2019a). We introduce in this study, the first model for exosomal release leveraging on *Aβ*-dependent intracellular *Ca*^2+^ homeostasis.

The article "A Neuron-Glial Model of Exosomal Release in the Onset and Progression of Alzheimer's Disease" was published in 2021. Journal: Front Comput Neurosci.

Our model design emphasizes a well-documented pathway for *Aβ* regulation of intracellular calcium that is amyloid-induced *Ca*^2+^ permeability through endogenous cation channels (Liu et al., 2010), such as L- and N-type voltage-gated calcium channels (VGCCs) and transient receptor potential melanostatin 8 (TRPM8) channels. These latter channels are prototypic temperature sensors and are emerging as possible key regulators in inflammation (Liu and Qin, 2011), often associated with Alzheimer's related neurodegeneration (Heppner et al., 2015).

This study is organized as follows. In section 2, we describe our model (the schematic representation of the model is given in Figure 1) in its different components: (i) *Ca*^2+^-dependent exosomal release in neurons and in astrocytes, (ii) astrocytic exosome exocytosis mediated by *Aβ* in AD, and (iii) temperature dependence of neuron models including *TRPM*8 currents. In section 3, we present numerical simulations based on the developed neuron-glial model. Finally, we discuss our results and outline future directions in section 4.

**Figure 1:** (Color online) The model astrocyte with different *Ca*^2+^ fluxes and *Ca*^2+^ signals. External stimulus triggers exosome release in calcium-dependent exocytosis. Astrocytic exosome exocytosis mediated by *Aβ* with the influence of the L-Type, T-Type, N-Type, and R-Type *Ca*^2+^ channels.

## 2. Methods

### 2.1. Calcium-Dependent Exosome Release in Neurons

The calcium-mediated exosomal release is restricted to active zones that contain VGCCs that control *Ca*^2+^ from the extracellular domain, mediate and regulate exocytosis, leading to the exosomal release in the brain (Veletić et al., 2020). This mechanism can be conveniently modeled by combining the Watts-Sherman model for *Ca*^2+^ exosomal release and the Montefusco-Pedersen models for *Ca*^2+^-regulated exocytosis, as originally put forth by Veletić et al. (2020). To link neuronal electrical activity and *Ca*^2+^-mediated exocytosis, we first describe intracellular *Ca*^2+^ dynamics, paying special attention to microdomain *Ca*^2+^ concentrations surrounding high-voltage activated L-type *Ca*^2+^ channels (*C*_*L*_) when the channels are opened (*C*_*L*|*opened*_) and closed (*C*_*L*|*closed*_), low-voltage activated T-type *Ca*^2+^ channels, as well as the characterization of *Ca*^2+^ below the plasma membrane (*C*_*m*_) in the bulk cytosol (*C*_*c*_), and in the endoplasmic reticulum (*C*_*r*_). In this fashion, exosomal release can be expressed as a function of L-type *Ca*^2+^ microdomain concentrations and plasma membrane *Ca*^2+^ concentrations, respectively, are as follows:


(1) $$\begin{array}{r} R_{C_{L}}=m_{C_{L}}^{2}h_{C_{L}}\cdot H\left(C_{L|opened},K_{L},n_{L}\right)+\left(1-m_{C_{L}}^{2}h_{C_{L}}\right)\\ \cdot H\left(C_{L|closed},K_{L},n_{L}\right), \end{array}$$

(2) $$\begin{array}{l} R_{C_{m}}=H\left(C_{m},K_{m},n_{m}\right), \end{array}$$

where $H\left(x,K,n\right)=\frac{x^{n}}{x^{n}+K^{n}}$ is the Hill function, *C*_*L*|*closed*_ = *C*_*m*_ (Montefusco and Pedersen, 2015), and the collective exosomal release rate in neurons is given by Veletić et al. (2020):


(3) $$\begin{array}{l} R_{n}=R_{C_{L}}+R_{C_{m}}. \end{array}$$

The whole-cell intracellular *Ca*^2+^dynamics ensues from the mass balance of *Ca*^2+^ fluxes across four different compartments: (i) *C*_*L*_; (ii) *C*_*m*_; (iii) *C*_*c*_ and (iv) *C*_*r*_. The equations for compartment-specific *Ca*^2+^ concentrations (Veletić et al., 2020):


(4) $$\begin{array}{l} \frac{dC_{L|opened}}{dt}=-f\left(\alpha \frac{I_{C_{L}}}{\lambda_{ud}}-B_{ud}\left(C_{L}-C_{m}\right)\right), \end{array}$$

(5) $$\begin{array}{r} \frac{dC_{m}}{dt}=\frac{f}{\lambda_{m}}(-\alpha I_{C_{T}}+N_{L}\Gamma m_{C_{L}}^{2}h_{C_{L}}\left(C_{L}-C_{m}\right)-\\ \lambda_{c}k_{PMCA}C_{m}-\lambda_{c}B_{m}\left(C_{m}-C_{c})\right), \end{array}$$

(6) $$\begin{array}{l} \frac{dC_{c}}{dt}=f\left(B_{m}\left(C_{m}-C_{c}\right)+p_{leak}\left(C_{r}-C_{c}\right)-k_{SERCA}C_{c}\right), \end{array}$$

(7) $$\begin{array}{l} \frac{dC_{r}}{dt}=\frac{f\lambda_{c}}{\lambda_{r}}\left(p_{leak}\left(C_{r}-C_{c}\right)-k_{SERCA}C_{c}\right), \end{array}$$

where the relevant parameters are provided in **Table 2**.

The article "A Neuron-Glial Model of Exosomal Release in the Onset and Progression of Alzheimer's Disease" was published in 2021. Journal: Front Comput Neurosci.

In terms of coefficients of the equations, *f* is the ratio of free-to-total *Ca*^2+^, Γ = λ_*ud*_*B*_*ud*_, α is the constant that transfers current to flux, *B*_*d*_ is the constant that defines the flux from the microdomains to the sub-membrane, the flux from the sub-membrane compartment to the bulk cytosol is defined by *B*_*m*_, while the volumes of a single microdomain, the sub-membrane compartment, the bulk cytosol, and the endoplasmic reticulum (*r*) are described by λ_*d*_, λ_*m*_, λ_*c*_, and λ_*r*_, respectively, *k*_*PMCA*_ is the rate of *Ca*^2+^ adenosine triphosphatase (ATPase) at the plasma membrane level, *p*_*leak*_ is the rate of the leak current from the *r* to the cytosol, and *k*_*SERCA*_ is the amount of *Ca*^2+^ sequestration into the *r* by the sarco/endoplasmic *Ca*^2+^ ATPase pump. The gating variables in the steady-state are defined in **Table 2**:


(8) $$\begin{array}{l} \frac{dm_{x}}{dt}=\frac{m_{x,\infty }\left(v_{m}\right)-m_{x}}{\tau_{mx\left(v_{m}\right)}};\frac{dh_{x}}{dt}=\frac{h_{x,\infty }\left(v_{m}\right)-h_{x}}{\tau_{hx\left(v_{m}\right)}}, \end{array}$$

where *x* = (*C*_*L*_, *C*_*T*_, *C*_*N*_, *Na, K*) and $B\left(x,v_{shift},v_{scale}\right)=\frac{1}{1+\exp\left(-\left(x-v_{shift}\right)/v_{scale}\right)}$.

The experimental evidence reveals that *Ca*^2+^-mediated exocytosis by neurons is regulated by intracellular *Ca*^2+^, where electrical activity pattern determines the exocytosis *Ca*^2+^ threshold (Pedersen et al., 2017). Electrical activity is triggered by neuron depolarization, which entails the activation of VGCCs, resulting in increased intracellular *Ca*^2+^concentration levels, which interfere with the mobilization of multivesicular bodies, resulting in the release of exosomes and evoking exocytosis (Shaheen et al., 2021). To describe the electrical activity of a depolarized neuron *via* membrane potential, we use the modified Hodgkin-Huxley neuron model, which includes voltage-gated potassium (*K*^+^) channels, voltage-gated sodium (*Na*^+^) channels, a leak current, and an induced control signal/current (*I*_*ind*_) as Veletić et al. (2020):


(9) $$\begin{array}{l} \frac{dv_{m}}{dt}=\frac{1}{c_{m}}\left(g_{K}\left(V_{K}-v_{m}\right)+g_{Na}\left(V_{Na}-v_{m}\right)+g_{L}\left(V_{L}-v_{m}\right)+I_{ind}\right), \end{array}$$

where *c*_*m*_ is the membrane capacitance, *V*_*K*_, *V*_*Na*_, and *V*_*L*_ are Nernst potentials for *K*^+^, *Ca*^2+^, and *Na*^+^ ions and other ions were clustered together as a “leak” channel, respectively, and *g*_*K*_, *g*_*Na*_, and *g*_*L*_ are the corresponding membrane conductances. The external stimulus *I*_*ind*_ is the current pulses of 500 ms with varying length and amplitude from 10 to 20 μA/cm^2^, voltage-gated conductances $(g_{K}=\bar{g_{K}}m_{K}^{4}$ and $g_{Na}=\bar{g_{Na}}m_{Na}^{3}h_{Na})$ fluctuate over time as action potentials are initiated and propagated (Shaheen et al., 2021).

### 2.2. Calcium-Dependent Exosomal Release From Astrocytes

Traditionally, astrocytes were thought to be non-excitable brain cells that only provided structural and metabolic support to neurons (Valenza et al., 2011). However, in the last two decades, this viewpoint has shifted and it has been revealed that astrocytes react to neurotransmitters and neuromodulators by increasing cytosolic *Ca*^2+^ concentration levels (Di Garbo et al., 2007). Indeed, a significant amount of experimental evidence, describing the signaling processes between astrocytes and astrocyte neurons, revealed the potential role of glial cells in neural tissue dynamics (Escartin et al., 2021; Wang et al., 2021). Astrocytes have glutamate-sensitive and metabotropic glutamate receptors (mGluRs) on their plasma membranes (Veletić et al., 2020). The glutamate initiates the intracellular release of *Ca*^2+^ ions from the endoplasmic reticulum triggered by mGluRs. This is accomplished by chemical reactions involving *IP*_3_, a secondary messenger molecule that is essential for *Ca*^2+^ mobilization into the cytosol. The *IP*_3_ synthesis has been defined simply in tripartite synapses (a term introduced to emphasize the existence of an astrocyte in the vicinity of two neurons), with the hypothesis that a quantized amount of *IP*_3_ molecules is released after glutamate levels rise due to pre-synaptic spiking activity (Veletić et al., 2019). We are interested in controlling *IP*_3_ with a defined stimulation pattern in our scenario, where the astrocyte differentiated from CNS functions as a neuron-independent unit. Therefore, the *IP*_3_ production rate (*P*), as a function of a generic control signal *v*_*ind*_ applied to depolarize the astrocyte, is given as follows (Veletić et al., 2020):


(10) $$\begin{array}{l} \frac{dP}{dt}=\frac{P_{0}-P}{\tau_{P}}+r_{P}. \end{array}$$

Next, combining (Equation 9) with *Ca*^2+^ dynamics we can propose a model with electrically silent astrocyte for *IP*_3_ development and *Ca*^2+^-dependent exocytosis. The *Ca*^2+^ dynamics surrounding L-Type and N-type *Ca*^2+^ channels delineate similarly to neurons. It is expected that L-type *Ca*^2+^- channels in neurons and astrocytes have identical qualities (Veletić et al., 2020). Hence, *C*_*L*_ concentration in a single astrocytic microdomains is epitomized in Equation (4) by setting *v*_*m*_ = *V*_*m*_ + *v*_*ind*_ in all corresponding equations, where *V*_*m*_ = −70*mV* gives the resting astrocytic membrane potential. The *Ca*^2+^ concentrations in single microdomains surrounding high-voltage activate N-type *Ca*^2+^ channels when the channels are opened and closed, and the plasma membrane (*C*_*m*_) lead to the following equations (Veletić et al., 2020):


(11) $$\begin{array}{l} \frac{dC_{N|opened}}{dt}=-f\left(\alpha \frac{i_{{Ca}_{L}}}{\lambda_{ud}}-B_{ud}\left(C_{N}-C_{m}\right)\right), \end{array}$$

(12) $$\begin{array}{l} \;\frac{dC_{m}}{dt}=\frac{f}{\lambda_{m}}(-\alpha i_{{Ca}_{T}}+N_{L}\Gamma m_{Ca_{L}}^{2}h_{Ca_{L}}\\ \left(C_{L}-C_{m}\right)-\lambda_{c}k_{PMCA}C_{m}-\lambda_{c}B_{M}\left(C_{m}-C_{c}\right)\\ +N_{N}\Gamma m_{Ca_{N}}h_{Ca_{N}}\left(C_{N}-C_{m}\right)), \end{array}$$

with *C*_*N*|*closed*_ = *C*_*m*_, where *i*_*C*_*N*__ = *g*_*C*_*N*__(*V*_*m*_ + *v*_*ind*_ − *V*_*C*_)/*N*_*N*_ and *g*_*C*_*N*__ is the membrane conductance of N-type *Ca*^2+^ channels. In modeling exosomal release from astrocytes, by manipulating the Nadkarni-Jung model that is further based on the Li-Rinzel model (Li and Rinzel, 1994) to define *Ca*^2+^ concentrations in the bulk cytosol and in the endoplasmic reticulum coupled in astrocytes, we have:


(13) $$\begin{array}{r} \frac{dC_{c}}{dt}=-c_{1}v_{1}m_{P,\infty }^{3}h_{P}^{3}\left(C_{c}-\frac{c_{0}-C_{c}}{c_{1}}\right)-c_{1}\\ v_{2}\left(C_{c}-\frac{c_{0}-C_{c}}{c_{1}}\right)-v_{3}\cdot H\left(C_{c},k_{3},n_{4}\right), \end{array}$$

where the values of parameters used in the above equations are given in Table 1 and the gating variable *m*_*P*,∞_ = H(*P, d*_1_, *d*_6_)·H(*C*_*c*_, *d*_5_, *d*_6_), *h*_*P*,∞_ = H(*Q, C*_*c*_, *d*_6_) adopted from Veletić et al. (2020), moreover


(14) $$\begin{array}{l} \frac{dh_{P}}{dt}=\frac{h_{P,\infty }-h_{P}}{\tau_{h_{P}}}, \end{array}$$

and *d*_6_ = 1, $\tau_{h_{P}}=\frac{1}{a_{2}\left(Q+C_{c}\right)}$, $Q=d_{2}\frac{P+d_{1}}{P+d_{3}}$. The *IP*_3_ molecules bind to receptors on the surface of the endoplasmic reticulum, allowing *Ca*^2+^ to be released once they are generated *in situ* (or obtained from other cells through gap junction). Since internal *Ca*^2+^ stores are also responsive to *Ca*^2+^, an increase in *Ca*^2+^ concentration deploys sufficient *Ca*^2+^ release. This biological process is known as Calcium-Induced Calcium Release (CICR) which shows the first term of Equation (12). Additional *Ca*^2+^ flow from the endoplasmic reticulum into the cytosol usually arises (leakage flow), while *Ca*^2+^ based ATPase pumps (SERCA) work in the opposite direction to uptake *Ca*^2+^ (second term of Equation 12) back into the stores for potential use (pump flow). The balance between passive leakage from the endoplasmic reticulum and SERCA uptake regulates *Ca*^2+^ concentration at rest. Sneyd and Li and Rinzel have identified analytically the *Ca*^2+^ dynamics and release/uptake processes triggered by *IP*_3_ (Escartin et al., 2021). Further, the relative exosomal release rate feature in astrocytes based on N-type *Ca*^2+^ microdomain concentrations, as Watts and Sherman did for glucagon secretion in pancreatic alpha cells (Watts and Sherman, 2014):


(15) $$\begin{array}{r} R_{C_{N}}=m_{C_{N}}^{2}h_{C_{N}}\cdot H\left(C_{N|opened},K_{N},n_{N}\right)+\left(1-m_{C_{N}}^{2}h_{C_{N}}\right)\\ \cdot H\left(C_{N|closed},K_{N},n_{N}\right). \end{array}$$

The relative exosomal release rate depending on *C*_*L*_, *C*_*m*_ concentrations that is, *R*_*C*_*L*__ and *R*_*C*_*m*__, follows Equations (1, 2), respectively, and the collective exosomal release rate in astrocytes is defined as follows (Veletić et al., 2020):


(16) $$\begin{array}{l} R_{a}=R_{C_{L}}+R_{C_{m}}+R_{C_{N}}. \end{array}$$

**Table 1:** Parameter set for calcium-mediated exosomal dynamics.

**Parameter**	**Value**	**Parameter**	**Value**	**Parameter**	**Value**
*V*_*K*_	−70(*mV*)	*V*_*L*_	−54.4(*mV*)	*V*_*h*_*C*_*T*___	−52(*mV*)
*V*_τ_*h*_*C*_*T*____	−50(*mV*)	*V*_τ_*m*_*C*_*T*____	−50(*mV*)	*V*_τ_*h*_*C*_*L*____	0(*mV*)
*V*_*m*_*C*_*T*___	−49(*mV*)	*V*_*h*_*C*_*L*___	−33(*mV*)	*V*_*m*_*C*_*L*___	−30(*mV*)
*V*_τ_*m*_*C*_*L*____	-23(*mV*)	*S*_*h*_*C*_*L*___	−5(*mV*)	*S*_*h*_*C*_*T*___	−5(*mV*)
τ_*m*0_*V*_*C*_*T*____	0(*ms*)	λ_*ud*_	2.62 × 10^−19^(*L*)	α	5 × 10^−15^(μ*molpm*/*As*)
λ_*m*_	5 × 10^−14^(*L*)	λ_*c*_	5.7 × 10^−13^(*L*)	*p*_*leak*_	3 × 10^−4^(*ms*^−1^)
*f*	0.01	τ_*m*_0__*V*_*C*_*L*____	0.05(*ms*)	*k*_*SERCA*_	0.100(*ms*^−1^)
*B*_*m*_	0.128(*ms*^−1^)	*g*_*L*_	0.3(*mS*/*cm*^3^)	*k*_*PMCA*_	0.300(*ms*^−1^)
*g*_*C*_*T*__	0.4(*nS*)	*g*_*C*_*L*__	0.7(*nS*)	*c*_*m*_	1(*uF*/*cm*^2^)
τ_*m*_*V*_*C*_*L*____	1(*ms*)	*K*_*m*_	2(*uM*)	*n*_*L*_	4
*n*_*m*_	4	*S*_*m*_*C*_*T*___	4(*mV*)	τ_*h*_0__*V*_*C*_*T*____	5(*ms*)
*S*_*m*_*C*_*L*___	10(*mV*)	*T*	10^*o*^*C*	*S*_τ_*m*_*C*_*T*____	12(*mV*)
τ_*m*_*V*_*C*_*T*____	15(*ms*)	*S*_τ_*h*_*C*_*T*____	15(*mV*)	*S*_τ_*m*_*C*_*L*____	20(*mV*)
*S*_τ_*h*_*C*_*L*____	20(*mV*)	τ_*h*_*V*_*C*_*T*____	20(*ms*)	$\frac{\lambda_{c}}{\lambda_{r}}$	31
$\bar{g_{K}}$	36(*mS*/*cm*^3^)	*V*_*Na*_	50(*mV*)	*K*_*L*_	50(μ*M*)
τ_*h*_0*V*_*C*_*L*____	51(*ms*)	τ_*h*_*V*_*C*_*L*____	60(*ms*)	*V*_*C*_	65(*mV*)
$\bar{g_{Na}}$	120(*mS*/*cm*^3^)	*N*_*L*_	200	*B*_*ud*_	264(*ms*^−1^)
*A*_*VL*_	1	*A*_*RYR*_	1	*A*_*m*_	1
*A*_*in*_	1	*l*	0.4, 1	*k*_1_	0.013
*k*_2_	0.18	*k*_*d*_	0.13	*n*_3_	3
*a*_1_	0.003	*a*_2_	0.02	*n*_5_	3.5
*n*_4_	2	λ_*PM*_	4.2	λ_*ast*_	3.49*1*e* − 13
*M*_*SERCA*_	15μ*M*/*s*	*M*_*CICR*_	10*s*^−1^	*M*_*PLC*_	0.05μ*M*/*s*
*M*_*PLC*_	0.05μ*M*/*s*	*n*_1_	2.02	*n*_2_	2.2
*P*_*SERCA*_	0.1μ*M*/*s*	*P*_*PC*_	0.3μ*M*/*s*	*P*_*CA*_	0.15μ*M*/*s*
*P*_*CI*_	0.15μ*M*	*c*_0_	2μ*M*	*P*_*IP*3_	0.1μ*M*
*P*_*deg*_	0.08*s*^−1^	*P*_*f*_	0.01*s*^−1^	ḡ_*T*_	0.0600*pS*
ḡ_*L*_	3.5000*pS*	ḡ_*N*_	0.3900*pS*	ḡ_*R*_	0.2225*pS*
*V*_*C*_	65*mV*	Δ*H*	−156*KJ*/*mol*	Δ*S*	−550*J*/*molK*
*z*	0.87	*R*	8.3144*J*/*molK*	*F*	96485*C*/*mol*
*c*_1_	0.185	*v*_1_	6*s*^−1^	*v*_2_	0.11*s*^−1^
*v*_3_	0.9μ*M*/*s*	*k*_3_	0.1μ*M*	*d*_1_	0.13
*d*_2_	1.049	*d*_3_	0.943	*d*_5_	0.082
*a*_2_	0.5/(μ*Ms*)	*IP*_30_	0.160μ*M*	*r*_*P*_	0.04μ*M*/*s*
τ_*P*_	1/0.000140*ms*	*V*_*m*_	−70*mV*	*g*_*C*_*N*__	0.6*nS*
*V*_*m*_*C*_*N*___	−5*mV*	*S*_*m*_*C*_*N*___	10*mV*	*V*_*h*_*C*_*N*___	33*mV*
*S*_*h*_*C*_*N*___	−5*mV*	τ_*m*_*V*_*C*_*N*____	1*ms*	τ_*m*_0__*V*_*C*_*N*____	0.05*ms*
*V*_τ_*m*_*C*_*N*____	−23*mV*	*S*_τ_*m*_*C*_*N*____	20*mV*	τ_*h*_*V*_*C*_*N*____	60*ms*
τ_*h*_0__*V*_*C*_*N*____	51*ms*	*V*_τ_*h*_*C*_*N*____	0*mV*	*S*_τ_*h*_*C*_*N*____	20*mV*
*N*_*N*_	200	*n*_*N*_	4	*K*_*N*_	2μ*M*

The article "A Neuron-Glial Model of Exosomal Release in the Onset and Progression of Alzheimer's Disease" was published in 2021. Journal: Front Comput Neurosci.

### 2.3. Amyloid-Beta Peptide Modulation of Astrocytic Exosome Exocytosis

Alzheimer's disease is one of the most prominent neurodegenerative diseases with an unknown structure of amyloid-beta peptide (*Aβ*). The distribution of *Ca*^2+^ astrocyte signaling plays an important role in AD. We have modified our previously elaborated model of *Ca*^2+^-mediated exosomal dynamics in neural cells to study spontaneous *Ca*^2+^oscillations in astrocytes in order to investigate the impact of *Aβ* on intracellular *Ca*^2+^ dynamics during AD. By activating the L-type VGCCs and metabolic glutamate receptors, or by increasing ryanodine receptor sensitivity and *Ca*^2+^leakage, *Aβ* will increase the resting concentration of intracellular *Ca*^2+^and adjust the regime of *Ca*^2+^ oscillations. The primary target of *Aβ* neurotoxicity is thought to be astrocytes (Gao et al., 2020). Astrocytes communicate with neurons and other brain cells in a functional way. Although astrocytes are not electrically excitable, they have a complex repertoire of intracellular *Ca*^2+^ signaling that changes across time and space within single astrocytes and through astrocytic networks (Semyanov et al., 2020). In an AD context, a computational model was recently used to investigate the effects of *Aβ* on *Ca*^2+^regulation (Latulippe et al., 2018).

In what follows, we provide further details of our new model to address the *Ca*^2+^-mediated exosomal release in astrocytes mediated by *Aβ* through four distinct pathways: VGCCs, metabotropic glutamate receptors 5, ryanodine receptor channels, and membrane leak (Gao et al., 2020). The *Aβ* deposit and its neurotoxicity associated with AD is involved in the disruption of *Ca*^2+^ regulation in astrocytes. Based on our previously discussed model, we have carried out a comprehensive simulation on *Ca*^2+^-mediated exosomal release in astrocytes mediated by *Aβ*, by also incorporating induced control signal/current. In the model of *Ca*^2+^-mediated exosomal release in astrocytes, different types of VGCCs are responsible for *Ca*^2+^ influx *J*_*VGCC*_ from the extracellular to the intracellular space. The Hodgkin-Huxley equations were used to describe the electrophysiological properties of these VGCCs and the related parameters are given in Tables 1, 2. Only the L-type VGCC current was thought to be mediated by *Aβ* in this study (Gao et al., 2020). All forms of *Ca*^2+^ ionic currents through VGCCs shared the simplified HH form:


(17) $$\begin{array}{l} I=gmh\left(v_{m}-V_{C}\right), \end{array}$$

where *g* represents membrane conductance, *m* and *h* represent the channel stimulation and inhibition (Zeng et al., 2009), respectively, whose values recover gradually to their steady-state values $\bar{m}$ and $\bar{h}$ given as


(18) $$\begin{array}{l} \frac{dy}{dt}=\frac{\bar{y}-y}{\tau_{y}}, \end{array}$$

where *y* = (*m, h*) and *v*_*m*_ is the membrane potential as given in Equation (9), *V*_*C*_ is the constant Nernst potential for calcium and other relevant parameters are given in Table 1 (Veletić et al., 2019, 2020; Gao et al., 2020).

The article "A Neuron-Glial Model of Exosomal Release in the Onset and Progression of Alzheimer's Disease" was published in 2021. Journal: Front Comput Neurosci.

**Table 2:** Details of voltage-gated calcium channels (VGCCs), time constants, and gating functions.

**Channel type**	**Equation of channel kinetics**
*m*_*K*/*Na*,∞_	$\frac{\alpha_{m_{K/Na}}}{\alpha_{m_{K/Na}}+\beta_{m_{K/Na}}}$
*h*_*Na*,∞_	$\frac{\alpha_{h_{Na}}}{\alpha_{h_{Na}}+\beta_{h_{Na}}}$
τ_*h*_*Na*__	$\frac{1}{\alpha_{h_{Na}}+\beta_{h_{Na}}}$
τ_*m*_*K*/*Na*__	$\frac{1}{\alpha_{m_{K/Na}}+\beta_{m_{K/Na}}}$
α_*m*_*Na*__	0.1(*v*_*m*_ + 40)B(*v*_*m*_, 40, 10)
β_*m*_*Na*__	4*exp( − (*v*_*m*_ + 65)/18)
α_*m*_*K*__	(0.01(*v*_*m*_ + 55))B(*v*_*m*_, 55, 10)
β_*m*_*K*__	0.125*exp( − (*v*_*m*_ + 65)/18)
α_*h*_*Na*__	0.07*exp( − (*v*_*m*_ + 65)/20)
β_*h*_*Na*__	B(*v*_*m*_, 35, 10)
*m*_*C*_*x*_,∞_	B(*v*_*m*_, *V*_*m*_*C*_*x*___, *S*_*m*_*C*_*x*___)
*h*_*C*_*x*_,∞_	B(*v*_*m*_, *V*_*h*_*C*_*x*___, *S*_*h*_*C*_*x*___)
*T*−*type*	*I*_*C*_*T*__ = ḡ_*T*_*m*_*T*_(*h*_*Tf*_ + 0.04*h*_*Ts*_)(*v*_*m*_ − *V*_*C*_)
	${\bar{m}}_{T}=B\left(v_{m},63.5,1.5\right)$
	${\bar{h}}_{Tf}=B\left(v_{m},76.2,3\right)$
	${\bar{h}}_{Ts}=B\left(v_{m},76.2,3\right)$
	$\tau_{h_{Tf}}=50*\exp\left(-{\left(\left(v_{m}+72\right)/10\right)}^{2}\right)+10$
	$\tau_{h_{Ts}}=400*\exp\left(-{\left(\left(v_{m}+100\right)/10\right)}^{2}\right)+400$
	$\tau_{m_{T}}=65*\exp\left(-{\left(\left(v_{m}+68\right)/6\right)}^{2}\right)+12$
*L*−*type*	*I*_*C*_*L*__ = ḡ_*L*_*m*_*L*_*h*_*L*_(*v*_*m*_ − *V*_*C*_)
	${\bar{m}}_{L}=B\left(v_{m},50,3\right)$
	${\bar{h}}_{L}=\left(0.00045/\left(0.00045+C_{c}/1000\right)\right)$
	$\tau_{m_{L}}=18\exp\left(-{\left(\left(v_{m}+45\right)/20\right)}^{2}\right)+1.5$
*N*−*type*	*I*_*C*_*N*__ = ḡ_*N*_*m*_*N*_*h*_N_*(*v*_*m*_ − *V*_*C*_)
	*m*_*N*_ = B(*v*_*m*_, 45, 7)
	*h*_*N*_ = 0.0001/(0.0001 + *C*_*c*_/1000)
	$\tau_{m_{N}}=18*\exp\left(-{\left(\left(v_{m}+70\right)/25\right)}^{2}\right)+0.3$
*R*−*type*	*I*_*C*_*R*__ = ḡ_*R*_*m*_*R*_*h*_*R*_((*v*_*m*_)−*V*_*C*_)
	${\bar{m}}_{R}=B\left(v_{m},10,10\right)$
	${\bar{h}}_{R}=B\left(v_{m},48,5\right)$
	$\tau_{h_{R}}=0.5*\exp\left(-{\left(\left(v_{m}+55.6\right)/18\right)}^{2}\right)+0.5$
	$\tau_{m_{R}}=0.1*\exp\left(-{\left(\left(v_{m}+62\right)/13\right)}^{2}\right)+0.05$
τ_*m*_*C*_*x*___	$\frac{\tau_{m_{V_{C_{x}}}}}{\exp\left(\frac{-\left(v_{m}-V_{\tau_{m_{C_{x}}}}\right)}{S_{\tau_{m_{C_{x}}}}}\right)+\exp\left(\frac{\left(v_{m}-V_{\tau_{m_{C_{x}}}}\right)}{S_{\tau_{m_{C_{x}}}}}\right)}+\tau_{m0_{V_{C_{x}}}}$
τ_*h*_*C*_*x*___	$\frac{\tau_{h_{V_{C_{x}}}}}{\exp\left(\frac{-\left(v_{m}-V_{\tau_{h_{C_{x}}}}\right)}{S_{\tau_{h_{C_{x}}}}}\right)+\exp\left(\frac{\left(v_{m}-V_{\tau_{h_{C_{x}}}}\right)}{S_{\tau_{h_{C_{x}}}}}\right)}+\tau_{h0_{V_{C_{x}}}}$

We use parameter *l* to reflect a fixed amount of *Aβ* concentration present in the environment to investigate the effects of *Aβ*. In addition, we use *A*_*VL*_ to monitor the strength of *Aβ* effects on the L-type VGCC current pathway, resulting in a total *Ca*^2+^current as follows:


(19) $$\begin{array}{l} I_{VGCC}=I_{C,T}+\left(1+A_{VL}l\right)I_{C,L}+I_{C,N}+I_{C,R}, \end{array}$$

where the corresponding flux is defined as


(20) $$\begin{array}{l} J_{VGCC}=-\frac{I_{VGCC}}{zF\lambda_{ast}}. \end{array}$$

The concrete formula for each type of calcium current is given in detail in Table 2 adopted from Zeng et al. (2009). The synthesis of *IP*_3_ catalyzed by phospholipase (PLC) is enhanced by cytoplasmic *Ca*^2+^ in this model. The *IP*_3_ receptors (*IP*_3_*R*) are mediated by cytoplasmic *Ca*^2+^ and *IP*_3_, inducing *Ca*^2+^ flow out of the endoplasmic reticulum by CICR. Importantly, CICR from the endoplasmic reticulum is perhaps the most well-studied *Ca*^2+^ signaling pathway in astrocytes (De Pittà et al., 2019). *Aβ* may mediate the L-type VGCC, metabotropic glutamate receptors 5 (mGluR5), ryanodine receptor (RyR) channels, and membrane leak *J*_*in*_ (Gao et al., 2020). Next, we define *J*_*SERCA*_ which represents the flux of calcium ions from the cytosol into the endoplasmic reticulum through the sarcoplasmic/endoplasmic reticulum calcium ATPase (SERCA). The leak flux due to the concentration gradient is indicated by the “leak” from the endoplasmic reticulum (*J*_*r*_). The other *Ca*^2+^fluxes *J*_*CICR*_, *J*_*SERCA*_, *J*_*RyR*_, *J*_*r*_, *J*_*in*_, and *J*_*pm*_ are defined as follows:


(21) $$\begin{array}{r} J_{CICR}=4M_{CICR}\cdot ℋ(P_{CA},C_{c},n_{1}).ℋ(C_{c},P_{CI},n_{1})\\ \cdot H(IP_{c},P_{IP_{3}},n_{2})((C_{r}-C_{c}) \end{array}$$

(22) $$\begin{array}{l} J_{SERCA}=M_{SERCA}\cdot H\left(C_{c},P_{SERCA},n_{4}\right), \end{array}$$

(23) $$J_{RyR}=(k_{1}+k_{2}\cdot H(C_{c},k_{d}+A_{RyR}l,n_{3})(C_{r}-C_{c}),$$

(24) $$\begin{array}{l} J_{r}=P_{f}\left(C_{r}-C_{c}\right), \end{array}$$

(25) $$\begin{array}{l} J_{in}=a_{1}+a_{2}P_{c}+A_{in}l^{n_{5}}, \end{array}$$

(26) $$\begin{array}{l} J_{pm}=\lambda_{PM}\cdot H\left(C_{c},K_{pm},n_{4}\right). \end{array}$$

In *J*_*in*_, *J*_*PLC*_, and *J*_*RyR*_, we also use *A*_*in*_, *A*_*RyR*_, *A*_*m*_ to monitor the intensity of these different effects, as well as *l* to represent the impact of *Aβ*. The essential parameters used in our analysis are listed in Table 1, they have been adopted from Gao et al. (2020). The modified *Ca*^2+^concentrations in the cytosol, endoplasmic reticulum, and the *IP*_3_ concentrations in the *IP*_*c*_ cell (*P*_*c*_) are defined as follows:


(27) $$\begin{array}{l} \frac{dC_{c}}{dt}=J_{VGCC}+J_{in}+J_{RyR}+J_{CICR}+P_{f}\left(C_{r}-C_{c}\right)-J_{SERCA}-J_{pm}, \end{array}$$

(28) $$\begin{array}{l} \frac{dC_{r}}{dt}=J_{SERCA}-J_{CICR}-J_{RyR}-P_{f}\left(C_{r}-C_{c}\right), \end{array}$$

(29) $$\begin{array}{l} \frac{dP_{c}}{dt}=J_{PLC}-P_{deg}P_{c}, \end{array}$$

where the initial concentrations are *C*_*c*_ = 0.1μ*M, P*_*c*_ = 0.1μ*M, C*_*r*_ = 1.5μ*M* at *t* = 0 motivated and validated by Gao et al. (2020) and *P*_*pC*_ is a half-saturation constant for calcium activation of *PLC*, *J*_*PLC*_ is the *IP*_3_ production rate and defined as:


(30) $$\begin{array}{l} J_{PLC}=\left(1+A_{m}l\right)M_{PLC}\cdot H\left(C_{c},P_{pC},n_{4}\right). \end{array}$$

In astrocytes, our model can replicate typical *Ca*^2+^ oscillations under the influence of *Aβ*. In addition, *Aβ*-containing exosomal release from astrocytes could be coupled by considering L-Type, N-type, and submembrane *Ca*^2+^ concentrations defined in Equations (4, 11–12). However, the bulk cytosol, endoplasmic reticulum, and *P*_*c*_ concentrations are the same as defined in Equations (27–29). Therefore, the relative exosomal release incorporating *Aβ* would be the same as defined in Equation (16) by using the concrete formula for each type of calcium current is given in Table 2. Further, we recall that, in astrocytes, transient elevations in cytoplasm-free *Ca*^2+^ levels can be thought of as a form of *Ca*^2+^ excitability (Valenza et al., 2011). The astrocytic plasma membrane contains a variety of neurotransmitter receptors, and experimental findings show that astrocytes near synapses react to neurotransmitters (such as glutamate, GABA, ATP, and others) by increasing their intracellular calcium levels (Di Garbo et al., 2007; Wang et al., 2012). The release of glutamate, ATP, and other neuromodulators substances is mediated by an increase in *Ca*^2+^, which can regulate synaptic communication between neurons through a biological process. Furthermore, recent studies show that glutamate produced by astrocytes influences neuronal activity by stimulating a depolarizing current in neurons (De Pittà, 2020). Therefore, for modeling the effect of glutamate release of astrocytes we used the Nadkarni and Jung model (Nadkarni and Jung, 2004) that considers a minimal neural network model made up of two coupled units: a pyramidal neuron and an astrocyte, by means of the *Ca*^2+^ concentration to the additional current toward the post-synaptic neuron:


(31) $$\begin{array}{l} I_{astro}=A_{astro}\cdot H\left[1000\cdot y\right]ln\left(y\right), \end{array}$$

where *y* = 1000 · *C*_*c*_ − 196.69, $A_{astro}=2.11\mu \text{A}/{\text{cm}}^{2}$, *H*(*x*) is the Heaviside function (Valenza et al., 2011) and *C*_*c*_ is the cytosolic calcium concentration in the astrocyte defined in Equation (27). Therefore, the modified membrane potential for the neuron-astrocyte network model is defined as follows (Di Garbo et al., 2007):


(32) $$\begin{array}{r} \frac{dv_{m}}{dt}=\frac{1}{c_{m}}(g_{K}\left(V_{K}-v_{m}\right)+g_{Na}\left(V_{Na}-v_{m}\right)\\ +g_{L}\left(V_{L}-v_{m}\right)+I_{ind}+I_{astro}). \end{array}$$

The article "A Neuron-Glial Model of Exosomal Release in the Onset and Progression of Alzheimer's Disease" was published in 2021. Journal: Front Comput Neurosci.

### 2.4. TRPM8 Channel Kinetics

In the present section, we will construct a more realistic neuronal model where the main characteristics account for temperature effects on *Ca*^2+^-dependant exosomal release in the neurons given in section 2.1. It is noteworthy to mention that in neurons potassium currents exceed sodium currents at higher temperatures, resulting in action potential failure. Thermal inhibition may, however, also be described by other temperature-dependent adjustments (Ganguly et al., 2019). Therefore, understanding the effects of temperature on *Ca*^2+^-mediated exosomal release could be very useful for a more precise design of strategies to control neural activity in the brain. We will use the modified Hodgkin-Huxley model to capture the response of *Ca*^2+^-mediated exosomal release in the neurons by varying the peak sodium and potassium conductances with temperature. It has been shown that the resting potential varies with the temperature (Ganguly et al., 2019). In the simplified neuronal model presented in section 2.1, the peak sodium and potassium conductances $\bar{g_{Na}}$ and $\bar{g_{K}}$, respectively, were considered to be constant and temperature independent as given in Table 1, but these values vary with temperature for a more realistic neuronal model, i.e., $(g_{K}=g_{Kmax}\left(T\right)m_{K}^{4}$ and $g_{Na}=g_{Namax}\left(T\right)m_{Na}^{3}h_{Na})$, where $g_{Kmax}\left(T\right)=1.60\exp^{-{\left(\frac{T-27.88}{12.85}\right)}^{2}}$ and $g_{Namax}\left(T\right)=0.42\exp^{-{\left(\frac{T-31.83}{31.62}\right)}^{2}}$ (Ganguly et al., 2019). Thus, while modeling the temperature effects, only the membrane potential, given in Equation (9), will be modified and the peak conductances values will be computed from the temperature-dependent gating variables defined as follows:


(33) $$\begin{array}{l} \{\begin{array}{l} \frac{dm_{K/Na}}{dt}=\phi_{m_{K/Na}}\left(T\right)\left(\alpha_{m_{K/Na}}\left(1-m_{K/Na}\right)-\beta_{m_{K/Na}}m_{K/Na}\right),\\ \frac{dh_{Na}}{dt}=\phi_{h_{Na}}\left(T\right)\left(\alpha_{h_{Na}}\left(1-h_{Na}\right)-\beta_{h_{Na}}h_{Na}\right), \end{array} \end{array}$$

where the functional dependencies of ϕ_*m*_*K*__, ϕ_*m*_*Na*__, and ϕ_*h*_*Na*__


(34) $$\begin{array}{l} \{\begin{array}{l} \phi_{m_{K}}\left(T\right)=4.3518\cdot 2.7^{\frac{T-20}{10}},\\ \phi_{m_{Na}}\left(T\right)=4.4288\cdot 3^{\frac{T-20}{10}},\\ \phi_{h_{Na}}\left(T\right)=3.8923\cdot 2.3^{\frac{T-20}{10}}, \end{array} \end{array}$$

are adopted from Ganguly et al. (2019) for the considered temperature of 25°C. Furthermore, we studied the somatosensory neuronal subset of cold thermosensors by creating a mathematical model of a cold sensing neuron in order to better understand the variety of ionic channels involved in *Ca*^2+^-dependent exosomal dynamics in neurons. Cold insensitive sodium channels are thought to play a role at extremely low temperatures, while TRPM8 has been established as a basic channel in characterizing cold-sensing neurons (Luiz et al., 2019). Voltage-gated potassium channels, in addition to these cold-specific ion channels, have been proposed to influence the temperature threshold degree of activation (Teichert et al., 2014). This model, in particular, shows how TRPM8 controls temperature-dependent initiation and inhibition at the threshold level. Note that a general Hodgkin-Huxley neuronal model is used here, with an additional current flowing through the TRPM8 channel (McGahan and Keener, 2020). Therefore, the modified membrane potential is defined as follows:


(35) $$\begin{array}{r} \frac{dv_{m}}{dt}=\frac{1}{c_{m}}(g_{K}\left(V_{K}-v_{m}\right)+g_{Na}\left(V_{Na}-v_{m}\right)\\ +g_{L}\left(V_{L}-v_{m}\right)+I_{ind}+I_{m8}). \end{array}$$

To give a current (*I*_*m*8_) for the cold sensing TRPM8 channel in contrast to the prior Hodgkin-Huxley model, prompted by McGahan and Keener (2020), with the current taking the following basic form:


(36) $$\begin{array}{l} I_{m8}=g_{m8}a_{m8}\left(v_{m}-V_{m8}\right), \end{array}$$

where *g*_*m*8_ is the maximal conductance of TRPM8 and *V*_*m*8_ is the reversal potential for TRPM8 channels. In addition, *a*_*m*8_ is temperature-dependent and given by Madrid et al. (2009) and McGahan and Keener (2020).


(37) $$\begin{array}{l} a_{m8}=B\left(\left(T+273.15\right)\Delta S,\Delta H-zFv_{m},R\left(T+273.15\right)\right), \end{array}$$

where Δ*H* and Δ*S* are the enthalpy and entropy variations in between closed and open states, respectively, *z* is the gating charge, *F* and *R* are Faraday's and universal gas constants, respectively, *T* is the temperature in ^*o*^C, and *V*_*m*8_, as previously stated, is the reversal potential of the TRPM8 channels, which has been experimentally shown to be near 0 *mV* (McGahan and Keener, 2020) and hence for all our analysis we set *V*_*m*8_ = 0. Furthermore, we will modify the neuronal model presented in section 2.3, where the main characteristics account for temperature effects on *Ca*^2+^-mediated exosomal release in astrocytes mediated by *Aβ*. To quantify the effects of temperature in the developed model, the membrane potential and the temperature dependant gating variables given in Equations (33–35) will be used. Moreover, we will develop a biologically driven model of a *Ca*^2+^-mediated exosomal release in astrocytes mediated by *Aβ* of a specific cold thermosensor with the existence of TRPM8 channels. Therefore, we couple the developed neuronal model with TRPM8 channels for analyzing the temperature threshold dependence on cold-sensing neurons, utilizing (Equations 35–37).

The article "A Neuron-Glial Model of Exosomal Release in the Onset and Progression of Alzheimer's Disease" was published in 2021. Journal: Front Comput Neurosci.

## 3. Results

### 3.1. Mechanism of *Ca*^2+^-Dependant Exosome-Release Both in Astrocytes and in Neurons

We start by quantifying the influence of *Ca*^2+^ mediated exocytosis on the membrane potential with a focus on microdomain *Ca*^2+^ concentrations around high-voltage activated L-type and low-voltage activated T-type *Ca*^2+^ channels. Also, a definition of *Ca*^2+^ below the plasma membrane, in the bulk cytosol, and in the endoplasmic reticulum using the *Ca*^2+^-mediated exosomal dynamics neuronal model. Moreover, the mechanism of *Ca*^2+^-dependant exosome release in response to square pulses of DC input currents of different amplitudes, both in neurons and astrocytes on the *Ca*^2+^-mediated exosomal dynamics is also investigated. The numerical results provided in this section are obtained by using the parameter values collected from Veletić et al. (2020), as presented in Table 1.

Motivated by Veletić et al. (2020), an external stimulus has been applied to excite the neurons by using the induced current pulses ranging from amplitudes of 10–20 μA/cm^2^ for a duration of 500 ms, as depicted in Figure 2A. The effects of the induced pulse of 10–20 μA/cm^2^ on the membrane potential have been presented in Figure 2B. As evident from this figure, the rate of generated sequences of the action potentials is proportional to both the magnitude and duration of the external stimuli. Not only this, but the spiking sequences are also significantly increased when the stimulus effect is incorporated within the numerical model. Importantly, these spiking sequences control the dynamics of the VGCCs in the membrane (Veletić et al., 2020). In addition, the rate of released exosomes from neurons with relative contributions of *Ca*^2+^ channels (evaluated by Equations 1–7) is shown in Figure 2C for the induced pulse of 10–20 μA/cm^2^. As evident from Figure 2C, the applied external stimulus increases action potential mediated oscillations around the baseline, resulting in a linear increase in exosomal release concentrations from neurons. As for astrocytes, the *IP*_3_ development rate is linearly proportional to the external stimuli *v*_*ind*_ adopted from Veletić et al. (2020).

The article "A Neuron-Glial Model of Exosomal Release in the Onset and Progression of Alzheimer's Disease" was published in 2021. Journal: Front Comput Neurosci.

**Figure 2:** (Color online) **(A)** Different amplitudes of induced control signals/currents ($I_{ind}\left(\mu \text{A}/{\text{cm}}^{2}\right)$) considered in the present study. **(B)** Responses/spiking sequence in the depolarized neurons, **(C)** the relative exosomal release rate in neurons, and **(D)** the relative exosomal release rate in astrocytes, for *I*_*ind*_ = 20 μA/cm^2^.

The corresponding exosomal release rate in astrocytes with relative contributions of the *Ca*^2+^ channels are evaluated by Equations (10–16) and is shown in Figure 2D corresponding to *v*_*ind*_ = 10 − 30 mV (Veletić et al., 2020), where one can approximate the release rate as constant during the controlling phase. It is noteworthy to mention that for the considered parameter set, the total concentration of exosomal release rate in astrocytes is mainly made up of concentrations based on N-type *Ca*^2+^ concentrations (for heavy depolarization), L-type *Ca*^2+^ concentrations, and sub-membrane *Ca*^2+^ concentrations (for weak depolarization). Astrocytes, unlike neurons, are electrically silent and incapable of generating action potentials (De Pittà and Berry, 2019b). This implies a variety of mechanisms, including chemical processes involving *IP*_3_, that cause astrocyte intracellular *Ca*^2+^ levels to rise. As shown in Figures 2C,D, these pathways have significantly slower dynamics than neuronal spiking, resulting in a significantly slower exosomal release by astrocytes as compared to the exosomal released by neurons. We detect an almost linear rise in the concentration of released exosomes from neurons for all stimuli intensities when non-depleted readily releasable exosomes are present in the cytosol throughout the stimulation period. We also found that three-quarters of the concentration of released exosomes in the considered scenario emanates from the concentration reliant on sub-membrane *Ca*^2+^ concentrations. As of exosomal release from astrocytes, we find that the concentration of released exosomes increases for all evaluated stimulus intensities when non-depleted readily releasable exosomes are present in the cytosol. Indeed, *Ca*^2+^ signaling is the most often observed readout of astrocyte activity in response to induced pulse, whether by synaptic activity, neuromodulators diffusing in the extracellular ambiance, or external chemical, mechanical, or visual stimuli. As shown by this interpretation, the individual astrocytic *Ca*^2+^ transient is viewed to some extent as an integration of the triggering external induced pulse and therefore is regarded as a demodulating of this pulse (De Pittà et al., 2019). It is worth noting that exosomes released by astrocyte activities demonstrated the capacity to specifically target neurons. Furthermore, the influence of the generated pulse/control signal presented in Figure 2A on the microdomain calcium concentrations is delineated in Figure 3. As evident, the increase in the amplitude of the control signal stimuli from 10 to 20 μA/cm^2^ results in a corresponding increase in the concentrations of *C*_*r*_, *C*_*m*_, *C*_*c*_, while the effect on the *C*_*L*_ concentration is quite negligible.

The article "A Neuron-Glial Model of Exosomal Release in the Onset and Progression of Alzheimer's Disease" was published in 2021. Journal: Front Comput Neurosci.

**Figure 3:** (Color online) Microdomain calcium concentrations: **(A)** *C*_*L*_, **(B)** *C*_*m*_, **(C)** *C*_*c*_, and **(D)** *C*_*r*_ corresponding to different values of control signals ranging from *I*_*ind*_ = 10 to 20 μA/cm^2^.

### 3.2. Characterization of Amyloid-Beta in Astrocytic-Calcium Signaling and Exosome Release

Calcium mediated exosomal release in astrocytes has been quantified for the membrane potential with particular attention given to microdomain *Ca*^2+^ concentrations surrounding L and T-type *Ca*^2+^ channels linked to a description of *Ca*^2+^ in the bulk cytosol, the endoplasmic reticulum, and the *P*_*c*_ concentrations. The numerical results presented in this section are based on the parameter values gathered (Ganguly et al., 2019; McGahan and Keener, 2020; Veletić et al., 2020) as presented in Tables 1, 2. This newly developed model aimed to explore the importance of VGCCs in astrocytic *Ca*^2+^-signaling and exosomal release mediated by *Aβ*. This study reproduced typical *Ca*^2+^ oscillations with the influence of *Aβ* (i.e., setting *l* = 0.4, 1) by integrating different types of VGCCs (Latulippe et al., 2018) in astrocytes. However, the four separate pathways mediated by *Aβ* (i.e., *VGCC*, *mGluR*5, *RyR*, and membrane leak *J*_*in*_) act to harm astrocytes by raising the frequency of *Ca*^2+^ oscillations, lowering the membrane threshold for *Ca*^2+^ oscillations, and enhancing the stable state concentration of *Ca*^2+^. Furthermore, by increasing *J*_*in*_, *Aβ* expands the membrane potential spectrum and raises resting *Ca*^2+^ concentrations to a low steady-state. The clustering of mGluR triggered by *Aβ* causes the oscillating range to change to a lower potential, as demonstrated in Gao et al. (2020). The increasing sensitivity of the *RyR* channel is primarily responsible for the amplitude of the *Ca*^2+^ oscillations. By triggering L-type *VGCC*, *Aβ* increases the resting *Ca*^2+^ at the high steady-state and moves the oscillating range to a lower potential. *Aβ* will activate L-type channels, resulting in an increase in intracellular *Ca*^2+^ concentration. We emphasize only the transition of *C*_*c*_ and *P*_*c*_ (defined in section 2.3) by applying an external stimulus presented in Figure 2A which has been applied to excite the neurons in the presence of *Aβ*. The effects of different values of *Aβ* on calcium concentrations for *C*_*c*_ and *P*_*c*_ without applying the induced/control signals stimulus is presented in Figure 4. It can be seen from Figure 4 that the simulated results and trends are fully consistent with the studies reported by Gao et al. (2020). It is observed that *Aβ* alters the membrane potential which in turn can enhance the regime of *Ca*^2+^ oscillations and increase the stable state concentration of *Ca*^2+^. The *Ca*^2+^ oscillations demonstrate that astrocytes have ionic excitability mediated by *Aβ*, making them possible targets for *Aβ* neurotoxicity. A pathological rise in *Aβ* may cause functional and structural abnormalities in glial cells, including *Ca*^2+^ dysregulation. This calcium/gliotransmission alteration might route a key component in the pathophysiology of AD. The calcium hypothesis of AD proposes that activation of the amyloidogenic pathway retrofits neuronal *Ca*^2+^ signaling, affecting normal *Ca*^2+^ homeostasis and the processes involved in learning and memory. Our results show that the presence of *Aβ* aggregates raises cytosolic *Ca*^2+^ levels. Exaggerated *P*_*c*_ concentrations evoked *Ca*^2+^ release with the influence of *Aβ* raises the amplitude of a *Ca*^2+^-activated hyperpolarizing current, which suppresses membrane excitability. Furthermore, as AD progresses, increasing the threshold for spike activation may have an effect on coincidence detection and local circuit activity. Additionally, the effect of the control signal presented in Figure 2A on the microdomain calcium concentrations has been depicted in Figure 5. It is evident from Figure 5 that the increase in the amplitude of the control signal stimuli from 10 to 20 μA/cm^2^ results in a corresponding increase in the concentration of *P*_*c*_ and *C*_*c*_. Cytosolic buffering determines the presence of a control signal across the plasma membrane in response to an increase in free cytosolic *Ca*^2+^ concentration, the rate of removal from the cytosol by sequestration into organelles (primarily *r*), and cell extrusion over the plasma membrane. Furthermore, external stimuli leverage subsequent *Ca*^2+^ influx by inactivating voltage- or receptor-operated channels in the bulk cytosol, activating *K* channels that lower membrane excitability, or influencing *Ca*^2+^ release from intracellular depots. The spatial distribution of *Ca*^2+^ signals is greatly influenced by cytosolic *Ca*^2+^ buffering. One of the major pathways for *Ca*^2+^ release from the endoplasmic reticulum is through *IP*_3_ receptors. The diffusion of *IP*_3_ concentration in the *IP*_*c*_ cell can stimulate *Ca*^2+^ release from the endoplasmic reticulum in response to the activation of the firing of action potentials by external stimuli. Increased concentrations of *P*_*c*_ pathways may then encourage the transition to a low-threshold activated L-type *Ca*^2+^ current, causing additional disturbance of intracellular *Ca*^2+^ homeostasis which is a key phenomenon for AD (Bertsch et al., 2020).

The article "A Neuron-Glial Model of Exosomal Release in the Onset and Progression of Alzheimer's Disease" was published in 2021. Journal: Front Comput Neurosci.

**Figure 4:** (Color online) Microdomain calcium concentrations for: **(A)** *C*_*c*_ and **(B)** *P*_*c*_ with the influence of *Aβ* (i.e., *l* = 0.4, 1) without induced/control signals.

**Figure 5:** (Color online) Microdomain calcium concentrations for: **(A)** *C*_*c*_ and **(B)** *P*_*c*_ corresponding to control signal shown in Figure 1A ranging as *I*_*ind*_ = 10–20 μA/cm^2^.

Furthermore, the *Ca*^2+^-dependant exosomal release from astrocytes in response to different representative values of extracellular *Aβ* has been presented in Figure 6 (Equation 16 used here and all relative equations found in sections 2.1, 2.2). As depicted in Figure 6, the relative contribution to *Ca*^2+^ signaling enhances the secretion of exosomal release in astrocytes from all components contributing to *Ca*^2+^ signaling in the cytoplasm (as defined in section 2.3). This means that astrocyte secretion will generate new synaptic connections for different values of *Aβ*, thus, increasing complexity of the neural network. Hence, increasing the values of *Aβ* would lead to a significant increase in the spiking sequence of exosomal release from astrocytes, while the effect on the concentrations of exosomal release rate is quite negligible. In addition, the effect of the control signal presented in Figure 2A on the *Ca*^2+^-dependent exosomal release from astrocytes has been presented in Figure 7 with and without the influence of activity-dependent *Aβ*. Figure 7 depicts that the exosomal release rate is substantially higher when the activity-dependent *Aβ* is involved in the model. The external stimulus enhances the influence of activity-dependent *Aβ* and the spiking sequences are significantly larger for the release of exosomes from astrocytes. The spiking sequences are also significantly reduced without the influence of activity-dependent *Aβ* as depicted in Figure 7.

The article "A Neuron-Glial Model of Exosomal Release in the Onset and Progression of Alzheimer's Disease" was published in 2021. Journal: Front Comput Neurosci.

**Figure 6:** (Color online) *Ca*^2+^-dependent exosomal release (μ M) from astrocytes corresponding to different values of *Aβ*, i.e., **(A)** *l* = 0.4 and **(B)** *l* = 1 without the influence of *I*_*ind*_.

**Figure 7:** (Color online) *Ca*^2+^-dependent exosomal release from astrocytes corresponding with and without the influence of activity-dependent *Aβ*, i.e., **(A)** *l* = 0 and **(B)** *l* = 0.4 with the influence of *I*_*ind*_.

Our findings suggest that *Aβ* enhances exosomal release from the astrocytes. Astrocytes, unlike neurons, are electrically quiet and cannot trigger action potentials. Because *Aβ* triggers astrocytes and neurophysiological properties of selected neurons by shifting from a high-threshold to a low-threshold triggered L-type *Ca*^2+^ current, this hints that a variety of pathways, including chemical processes involving *Aβ*, cause an increase in astrocyte intracellular *Ca*^2+^ levels. It could be an underlying mechanism for the early metabolic and noncognitive symptoms of AD caused by hypothalamic dysfunction.

### 3.3. Characterization of Neural Activity in the Presence of Exosomal Release From Astrocytes

In this section, we will discuss the dynamics of neural activity in the presence of exosomal release from astrocytes by analyzing it with a model involving an astrocyte coupled to a single neuron, as developed in section 2.3. The biological processes involving astrocytes take place in close proximity to the synapses of neurons. They are sensitive to neuronal activity sensors that react to glutamate synaptic release with oscillations in intracellular calcium concentration. The concentration of *P*_*c*_ is triggered by glutamate elevations in the astrocyte domain, which activates intracellular *Ca*^2+^ dynamics. The amplitude, frequency, and propagation of intracellular *Ca*^2+^ oscillations produced in astrocytes are regulated by the intrinsic properties of both neuronal inputs and astrocytes. Astrocytes can distinguish between numerous forms of neuronal inputs and incorporate concomitant inputs in response to calcium elevations. Calcium dynamics are regulated by the interaction of CICR, which is a nonlinear amplification mechanism dependent on calcium channels opening to calcium stores, such as the endoplasmic reticulum. The action of active transporters causes a reverse flow (SERCA pumps). Signals impinging on the cell from an outside environment directly regulate the level of *P*_*c*_ (De Pittà, 2020). As a result, the calcium signal can be viewed as encoded information about the intensity of *P*_*c*_. The release of glutamate from the astrocyte is triggered by an increase in intracellular calcium levels in astrocytes, which promotes a depolarizing current in neurons (*I*_*astro*_), modulating pre-synaptic and post-synaptic neural activities. When a neuron fires, small quantities of neurotransmitters (glutamate) are released into the synaptic cleft. The release of intracellular *P*_*c*_ is triggered when neurotransmitters bind to glutamate receptors on astrocytes. The action potentials generated by the neuron injected with a constant current *I*_*ind*_, trigger an increase of the internal *Ca*^2+^ concentration of the astrocyte. This event feedbacks an inward current to the neuron (*I*_*astro*_).

The article "A Neuron-Glial Model of Exosomal Release in the Onset and Progression of Alzheimer's Disease" was published in 2021. Journal: Front Comput Neurosci.

The time course of the membrane potential and cytosolic *Ca*^2+^ concentrations in the presence of exosomal release from the astrocyte, when the neuron is injected with the current *I*_*ind*_ = 20 μA/cm^2^, are presented in Figure 8. The results presented in Figure 8 show that the generation of firing activity in the exosomal release from neurons occurs during the stimulation phase alone. In this case, the elevation of the internal *Ca*^2+^ level in the astrocyte is not sufficient to trigger a feedback response in the neurons (see Equation 32). The increase of the production rate of *P*_*c*_ amplifies the *Ca*^2+^ response in the astrocyte and so leads to the generation of membrane potentials within a well-defined time window. The neural dynamics of membrane potential (*v*_*m*_ given in Equation 32) and *C*_*c*_ are altered by the surrounding activity, i.e., the astrocyte feedback. To illustrate the impact of the astrocytic feedback on neural excitability, we study the neural activity dynamics generated by our model both with and without *Aβ*. Numerical simulations of dynamical regimes in which neuronal firing is sustained indefinitely revealed that cytosolic *Ca*^2+^ concentration and membrane potential fluctuate rapidly under the control of *Aβ* while spiking sequences are greatly decreased when *Aβ* is not present (Figure 8). This pattern of activity is symptomatic of strong excitability of the neuronal system that can turn into hyperexcitability during a pathological crisis. In the time series generated by the model without *Aβ* (Figures 8A,C), the neural activity and the glutamate concentration dynamics remain unchanged after the instantaneous increase of *I*_*ind*_ = 20 μA/cm^2^, which mimics glutamate release. In contrast, in the model with *Aβ* i.e., *l* = 0.4 (Figures 8B,D), the strong increase in the spiking sequences of membrane potential and *C*_*c*_ enhance the glutamate release that halts neuronal activity. Once the action potentials have become sufficiently low, neural activity re-emerges and glutamate and concentrations come back to their respective basal values, oscillating with neural activity. Our results imply that neuronal activity controls the regional sensitivity of *Aβ* formation. Although much of this discussion focuses on *Ca*^2+^-regulated exosomal release from astrocytes in the presence of *Aβ*, we cover one transporter, in particular, the cystine/glutamate transporter, because it is important in neurodegenerative disorders, such as AD. Cytosolic *Ca*^2+^-regulated glutamatergic gliotransmission activates neuronal extrasynaptic NMDA receptors, altering neuronal excitability and regulating synaptic transmission. Our findings point to a mechanism that might explain why neuronal activity in AD is susceptible to *Aβ* deposition.

The article "A Neuron-Glial Model of Exosomal Release in the Onset and Progression of Alzheimer's Disease" was published in 2021. Journal: Front Comput Neurosci.

**Figure 8:** (Color online) Behavior of membrane potential corresponding to *Aβ* **(A)** *l* = 0, **(B)** *l* = 0.4, and *C*_*c*_ **(C)** *l* = 0, **(D)** *l* = 0.4 with *I*_*ind*_ = 20 μA/cm^2^.

### 3.4. Temperature Dependence, With Emphasis on TRPM8-Mediated Modulations of Membrane Potential

The excitability and response characteristics of a neuron might change depending on the temperature of the surroundings. The effects of the induced pulse of 20 μA/cm^2^ on the membrane potential with temperature (*T* = 25 °C) and without the temperature effects have been presented in Figure 9. As evident from Figure 9, the pace of produced sequences of action potentials is proportional to both the amplitude and length of the external stimuli. Not only that, but when temperature effects are included in the numerical model, the spiking sequences are considerably decreased. Importantly, these spiking sequences regulate the kinetics of VGCCs in the membrane (Veletić et al., 2020). Variations of membrane potential have been observed when the membrane temperature is increased/decreased, indicating that the cell membrane environment in neurons becomes more electronegative/electropositive. The amplitude of action potentials, defined as the voltage difference between the threshold and the peak, and their duration, assessed by the breadth of the action potential at the threshold, were both impacted by temperature changes.

The article "A Neuron-Glial Model of Exosomal Release in the Onset and Progression of Alzheimer's Disease" was published in 2021. Journal: Front Comput Neurosci.

**Figure 9:** (Color online) The effect of temperature on the responses/spiking sequence in the depolarized neurons for *I*_*ind*_ = 20 μA/cm^2^.

The effects of the temperature on the microdomain calcium concentrations have been presented in Figure 10. As seen from the analysis of this figure, the intracellular *Ca*^2+^ concentrations in the closed and open channels of L-type, plasma membrane, bulk cytosol, and endoplasmic reticulum are significantly overestimated if the effect of temperature is neglected and the spiking sequences are also significantly reduced. Indeed, incorporating temperature will result in a corresponding decrease in the concentration of *C*_*r*_, *C*_*m*_, *C*_*c*_, and *C*_*L*_ concentrations, and the spiking sequences are also significantly reduced. The findings underpin Huxley's theory that thermally induced block is caused by increased activation of voltage-dependent potassium ion channels in response to depolarization, particularly at higher temperatures (Ganguly et al., 2019). The membrane depolarizes in response to depolarizing currents produced by an advancing action potential. The voltage-dependent potassium ion channels are activated, allowing potassium ions to flow out of the neuron, hyperpolarizing it. The depolarizing current that triggered these channels is antagonized by the hyperpolarizing current that passes through them. As a result, this process efficiently and quickly stops the action potential from propagating. Since depolarizing current forms an advancing action potential, a hyperpolarizing current is more powerful than simply blocking all ion channels. Instead of being actively antagonized, this action potential will spread through the passive region of blocked ion channels, diminishing only as it leaked out through the passive components of the neuronal membrane, such as leak channels and capacitance. Moreover, the exosomal release rate in neurons is directly linked with the *Ca*^2+^ concentrations in different compartments. The exosomal release rate is relatively higher when temperature effects are incorporated within the model. This can be attributed to the fact that an increase in temperature values will lead to a corresponding increase in the net hyperpolarizing current. The sodium inward current became shorter and the potassium outward current became faster and larger due to the increased speed of sodium/potassium ions gated conductances. As the membrane was depolarized by the action potential, the net current in the neural network became steadily outward (hyperpolarizing) with increased temperature which enhances neural activity. Thus, the exosomal release rate of the targeted neuron is significantly affected by the changes in temperature.

The article "A Neuron-Glial Model of Exosomal Release in the Onset and Progression of Alzheimer's Disease" was published in 2021. Journal: Front Comput Neurosci.

**Figure 10:** (Color online) Microdomain calcium concentrations: **(A)** L-Type *Ca*^2+^ concentration, **(B)** Sub-membrane *Ca*^2+^ concentration, **(C)** Cytosolic *Ca*^2+^ concentration and **(D)** Endoplasmic reticulum *Ca*^2+^ concentration with (red color) and without (black color) temperature effects corresponding to control signal of $I_{ind}=20\mu \text{A}/{\text{cm}}^{2}$.

Next, considering the state of cold sensing neurons we added the TRPM8 component in the present model by making *g*_*m*8_ nontrivial (i.e., *g*_*m*8_ = 3). We begin by using (Equation 36) of TRPM8 channels at different physiological voltages in response to temperature. Figure 11 represents the variation of the TRPM8 current in response to temperature and voltage. We combined the Equation (36) of TRPM8 channels with the induced control signals/currents stimulation given in Figure 2A that helps describe the overall behavior of *Ca*^2+^ concentrations at different temperature levels (see Equation 35). From Figure 11 we observe that as the fixed temperature level is raised, a few distinct characteristics occur. The stimulation-induced control signals/currents show decreasing amplitudes of the action potentials as the maximum voltage achieved for *Ca*^2+^ concentrations decreases with rising temperatures. Additionally, as the temperature rises, the average amplitude of the TRPM8 current grows. We should recognize that since *V*_*m*8_ = 0 (McGahan and Keener, 2020), the TRPM8 current will flow both inward and outward depending on the membrane potential, nonetheless, it is worth noting that at temperature effects ranging from *T* = 5 to 15°C there is an increase in outward current and concentration of *C*_*r*_, *C*_*m*_, *C*_*c*_, and *C*_*L*_ that behave differently corresponding to each temperature prescribed in Figure 11. The amplitude of the action potential decreases and its duration decreases as the temperature rises. The temperature dependence of ion channel conductance as well as the time constants of channel activation/inactivation factors may have an effect on neuronal function. Thus, temperature variations significantly affect the *Ca*^2+^ concentrations, the rates of diffusion, the rates of conformational changes, and the rates of metabolic processes. Similarly, as before, it is seen that an increase in temperature will result in a corresponding increase in the concentrations of *C*_*r*_, *C*_*m*_, and *C*_*c*_ while the effect on *C*_*L*_ concentrations is quite negligible. The scenario considered in this study is the presence of cold neurons affecting the concentrations of *Ca*^2+^-dependent exosomal release in neurons defined in section 2.1.

The article "A Neuron-Glial Model of Exosomal Release in the Onset and Progression of Alzheimer's Disease" was published in 2021. Journal: Front Comput Neurosci.

**Figure 11:** (Color online) Microdomain calcium concentrations for: **(A)** L-Type *Ca*^2+^ concentration, **(B)** Sub-membrane *Ca*^2+^ concentration, **(C)** Cytosolic *Ca*^2+^ concentration and **(D)** Endoplasmic reticulum *Ca*^2+^ concentration corresponding to control signal of $I_{ind}=20\;\mu \text{A}/{\text{cm}}^{2}$ and *I*_*m*8_ for different values of temperature.

Examining the behavior of the established model as *g*_*m*8_ is increased in response to the simulated temperature ramp shown in Figure 12A is also instructive. There are two consistent features across the three different values of *g*_*m*8_, as well as one that emerges as *g*_*m*8_ is increased. In Figure 12, we observe that when the neuron turns on and off, there are large amplitude jumps in the oscillations of membrane potential. Furthermore, in each of the Figures 12B–D, the neural activity is asymmetric on the down and up to temperature ramps, with the oscillations on the up temperature ramp lasting longer. Finally, when *g*_*m*8_ is increased, the neuron stops oscillating in the coldest part of the temperature ramp. The oscillations shrink in amplitude as the neuron is osed to lower temperatures, as seen in the plots with *g*_*m*8_ = 5 and *g*_*m*8_ = 10. While these voltage-time plots provide an overview of the role of TRPM8 channels in neuron activation and inactivation, they do not provide a complete picture. In particular, in the absence of induced control signals/currents, we wish to include a more complete description of the interactions between each of the ionic currents and temperature. The temperature ramp simulation with increasing TRPM8 maximal conductance provides a better picture of what the neurons are subjected to physiologically. The temperature-induced scaling of the rate constants, on the other hand, can have a significant impact on the length of the action potential. Temperature impacts the rate of neuron firing as well as the pace of action potential propagation. Variations in action potential frequencies with temperature are related to changes in resting potentials, but not in a straightforward manner. Cooling lowers the resting potential (depolarization), which leads to a rise in action potential frequencies, yet, when the temperature is increased, certain nerve cells exhibit an increase in frequency.

**Figure 12:** (Color online) Membrane potential in response to an external temperature ramp. The periodic spiking activity of the neuron in response to temperature ramp **(A)** plotted against time with: **(B)** *g*_*m*8_ = 3, **(C)** *g*_*m*8_ = 5, and **(D)** *g*_*m*8_ = 10.

The article "A Neuron-Glial Model of Exosomal Release in the Onset and Progression of Alzheimer's Disease" was published in 2021. Journal: Front Comput Neurosci.

The effects of the induced pulse of 20 μA/cm^2^ on the cytosolic calcium and the *IP*_3_ concentrations in the *IP*_*c*_ cells in regards to astrocytic exosome exocytosis mediated by *Aβ* in AD (see section 2.3), with temperature (*T* = 25°C) and without the temperature effects have been presented in Figures 13A,B. The kinetics of *C*_*c*_ and *IP*_3_ was markedly accelerated by increasing temperature. At *T* = 25 ^*o*^C, Figures 13A,B show that the rate of exosomal release of the astrocytes is proportional to both the magnitude and duration of the temperature and external stimuli. Therefore, increasing temperature will reduce the spiking sequences which enhance neural firing or promote neural activity. The temperature may increase exosomal release from neurons and glial cells, contributing to *Aβ* accumulation and hyperexcitability. The effect of temperature has been examined on cytosolic *Ca*^2+^ concentrations and the *IP*_3_ concentrations mediated by *Aβ*. Importantly, *Ca*^2+^ wave propagation is thought to be a reaction/diffusion system requiring several cycles of *Ca*^2+^ release from *IP*_3_ clusters and diffusion to nearby clusters to trigger CICR. The study found that the concentrations of *Ca*^2+^ and *IP*_3_ in the *IP*_*c*_ cells decrease monotonically with temperature which disturbs the brain dynamics and could lead to the pathophysiology of AD.

**Figure 13:** (Color online) Microdomain calcium concentrations for **(A)** *C*_*c*_, **(B)** *P*_*c*_, with and without temperature effects corresponding to control signal shown in Figure 2A.

Moreover, a study has been conducted to quantify the effects of TRPM8 channels in the modeling of *Ca*^2+^-mediated astrocytic exosome exocytosis mediated by *Aβ* (*l* = 0.4) in AD. The TRPM8 part of the model is added by setting *g*_*m*8_ to nonzero. The open possibility of TRPM8 channels, *a*_*m*8_, in response to temperature at various physiological voltages is first added. All other parameter values are set to Hodgkin-Huxley norms and *g*_*m*8_ = 3. As the fixed temperature level is raised, a few distinct features emerge that include the amplitudes of the action potentials increase, resulting in an increase in the maximum voltage reached. As a result, the current model emphasizes the importance of TRPM8 channels in determining temperature-dependent activation and inactivation thresholds. Furthermore, our findings shed light on what happens at the temperature levels at which these neurons shut down, as well as the role sodium and leak currents can play. It has been demonstrated by using both TRPM8 and the stimulus of induced control signal triggered the calcium concentrations of *C*_*c*_ and *P*_*c*_ defined in (Equations 27, 29). From Figures 14A,B, as the fixed temperature level is increased, a few distinct characteristics emerge in the presence of cold sensing neurons TRPM8 channels. The simulation shows that as the temperature rises, the amplitudes of the action potentials decrease as the maximum concentration of *C*_*c*_ and *P*_*c*_ declines. It can be seen from Figures 14A,B that increasing temperature from *T* = 5 to 15°C would result in a corresponding decrease in the concentration of *C*_*c*_ and *P*_*c*_ in the presence of *g*_*m*8_ = 3. However, TRPM8 channels were shown to be expressed in the endoplasmic reticulum where their modulation by activators and/or inhibitors was demonstrated to be crucial for intracellular *Ca*^2+^ signaling. The rise in inward flux is primarily responsible for the shift in the TRPM8 current amplitude, in fact, it is worth noting that from *T* = 5 to 15°C there is an increase in outward current. These findings imply that TRPM8 channels confer temperature sensitivity to the endoplasmic reticulum, which permits *Ca*^2+^ release by facilitating *Ca*^2+^ efflux into the cytosol and therefore contributing to CICR *via* *IP*_3_ and ryanodine receptors. Although the *IP*_3_ evoked *Ca*^2+^ signals were qualitatively comparable at 5–15 *Ca*^2+^, this difference in temperature should take into account the temperature sensitivity of *IP*_3_-mediated signal amplitudes. The transition temperature was 25°C in all cases, which might indicate a phase change in the lipids of the cytoplasmic membrane. Our findings demonstrate that using this temperature range (from *T* = 5 to 15°C) significantly increases the amplitude and lowers the frequency of global *IP*_3_-mediated *Ca*^2+^ signals, which is consistent with findings from a variety of different cell types. For instance, fast cooling elicits strong oscillatory *Ca*^2+^-activated leak currents when the *IP*_3_ pathway is active and has been shown to enhance the amplitudes of *IP*_3_-mediated *Ca*^2+^ signals in several cultured glial cells, including Schwann cells and olfactory ensheathing cells, as well as astrocytes. As a result, the temperature sensitivity of the cytosolic *Ca*^2+^ concentration underpinning global *IP*_3_-mediated signals appears to be a common occurrence, which must be taken into account when extending data obtained at room temperature to body temperature.

The article "A Neuron-Glial Model of Exosomal Release in the Onset and Progression of Alzheimer's Disease" was published in 2021. Journal: Front Comput Neurosci.

**Figure 14:** (Color online) Microdomain calcium concentrations for **(A)** *C*_*c*_, **(B)** *P*_*c*_ corresponding to *I*_*m*8_ and control signal shown in Figure 2A for different values of temperature, in presence of *Aβ*.

## 4. Conclusion and Discussion

We presented an integrated mathematical model for therapeutic exosomal release modulated by an externally applied stimulus. The proposed model combines cell activation, intercellular signaling, and exocytosis and allows to shed light on the relative roles of different subcellular *Ca*^2+^ compartments and astrocytes in exosomal release regulation. We implemented a novel model for accurately quantifying the *Ca*^2+^-mediated astrocytic exosome exocytosis mediated by amyloid-beta in AD. In addition, a comparative analysis has been conducted to quantify the effect of temperature and cold-sensitive neurons on the *Ca*^2+^-dependent exosomal release mediated by VGCCs and amyloid-beta in AD. Moreover, we calculated the astrocytic current as a function of both the pre-synaptic neuron current and the astrocyte (Li-Rinzel model). This work describes the synapse and astrocyte couplings in a computationally efficient model. It is possible to simulate real-time spiking artificial neuron-glia networks using the model proposed in this study, revealing the mechanism that appears to be a necessary part of the regulation of spiking activities. We showed that this model can be used to simulate the neuron astrocyte interaction. The results obtained with the developed model suggest that cell depolarization in neurons is directly related to the exosomal release which is proportional to the applied stimulation. The novelty of the present research is in the development of the *Ca*^2+^-mediated exosomal dynamics model of neurons accounting for the temperature effects with emphasis on TRPM8-mediated modulations of membrane potential. Further, it has been observed that *Ca*^2+^ concentrations in the respective compartments, and thus the overall *Ca*^2+^-mediated exosomal dynamics are significantly affected by the changes in temperature and TRPM8 channels. The findings show that TRPM8 and VGCCs play an important role in determining temperature-dependent activation and inactivation at numerous threshold levels. Thermal effects caused by cold detecting neurons cause *Ca*^2+^ to be released from the endoplasmic reticulum of primary spiral ganglion neurons. The activation of TRPM8 channels causes *Ca*^2+^ release, which is amplified by CICR. TRPM8 channel that colocalizes with the endoplasmic reticulum, is immunostained in the neurons. Indeed, the original and modified Hodgkin/Huxley models have a high degree of qualitative agreement, and the findings of this study are a significant move toward a better understanding of a novel modality for altering neural activity. The developed neuronal model provides an important step not only for our better understanding of the exosomal dynamics in neurons and astrocytes but also paves the way for the generation of new models aiming at optimizing and designing exosome-based drug delivery systems for the treatment of brain pathologies and neurodegenerative disorders such as AD.

The article "A Neuron-Glial Model of Exosomal Release in the Onset and Progression of Alzheimer's Disease" was published in 2021. Journal: Front Comput Neurosci.

Our model supports the view that astrocytes normally serve as neuronal signaling events, but in AD, they transform into astrocyte-derived exosomes, which can disrupt neurons *via* unknown mechanisms (Goetzl et al., 2016). The development of methods for isolating *Ca*^2+^-dependent exosome-release both in astrocytes and neuronally derived exosomes from plasma has enabled researchers to quantify neuronal proteins important in the pathogenesis of human neurodegenerative diseases. The astrocyte-derived exosomes were shown to be positive for neuroglobin, a protein that acts as a neuroprotectant against cell injury (Venturini et al., 2019); the notion that exosomes transmit neuroglobin to neurons would add another mechanism to the possible astrocytic neuroprotectant activity. Control signal microdomain *Ca*^2+^ concentrations unavoidably impact a wide range of neuronal activities, from the regulation of the overall cytosolic *Ca*^2+^ signal to the production of cell death. Multiple changes in this particular signaling pathway are prevalent in several neurodegenerative disorders, including AD, PD, and amyotrophic lateral sclerosis (ALS), emphasizing its importance. To further substantiate our findings presented on this study, a variety of future investigations into the astrocyte sources and cytotoxic mechanisms of complement proteins in astrocyte-derived exosomes will be needed. However, the definitive etiological relationships between the neuronal accumulation of primary neurotoxic proteins such as amyloid-beta, tau, and reductions in synaptic proteins that contribute to early synaptic dysfunction are now being discovered (Goetzl et al., 2018). It is worth noting that changes in intracellular *Ca*^2+^ signaling decrease neuronal interactions and enhance both acute and chronic degenerative diseases of the nervous system. In the present study, we found that due to the biophysical properties of voltage-gated and ligand-activated ion channels and receptors, *Ca*^2+^ fluxes through the neuronal membrane are strictly time-constrained. The neural activity could be enhanced by *Ca*^2+^-dependent receptors and channels, constantly rearranged as they are embedded in the crowded dynamic environment of biological membranes, allowing for temporary interaction and the creation of transient signals. In a highly dynamic environment, efficient *Ca*^2+^-mediated signal transduction necessitates mechanisms that support the very precise spatiotemporal alignment of the *Ca*^2+^ source and *Ca*^2+^-dependent exosomal exocytosis (De Pittà, 2020). Neuroprotective strategies that target various aspects of the dynamic regulation of intracellular *Ca*^2+^ signaling are a promising avenue for pharmaceutical intervention in nervous system neurodegenerative diseases, such as AD. Moreover, several intracellular *Ca*^2+^ signaling regulators found on the plasma membrane and intracellular organelles have been implicated in many of these pathophysiological processes (Valori et al., 2019). Our current understanding sheds new light on the essential roles of *Ca*^2+^ channels in synapse formation and function in the healthy central nervous system. Importantly, the previous studies were focused on the effect of temperature and TRPM8 channels on *Ca*^2+^-dependent exosome-release, where the temperature has been linked to dementia and may play a role in clinical phenotypes, particularly in the frontotemporal lobar degeneration continuum, but the cause of these symptoms has yet to be determined (Fletcher et al., 2015; De Pittà and Berry, 2019b; McGahan and Keener, 2020). Furthermore, altered neural activity and temperature perceptions may be expected in some neurodegenerative disorders, including AD, that can lead to impairments of the integrity of distributed and temperature processing networks. Alzheimer's syndrome is a notable test case. Future studies will be focused on the inclusion of other *Ca*^2+^ compartments linked to the integration of experimental mice model data of AD and on the development of a new stochastic model based on the ideas highlighted in this study.

The article "A Neuron-Glial Model of Exosomal Release in the Onset and Progression of Alzheimer's Disease" was published in 2021. Journal: Front Comput Neurosci.

## Data Availability Statement

The raw data supporting the conclusions of this article will be made available by the authors, without undue reservation.

## Author Contributions

HS: methods and materials, data curation, formal analysis, investigation, writing, and original draft preparation. SS and RM: designed research. SS: methodology, formal analysis, writing, review and editing, and supervision. RM: conceptualization, supervision, and reviews. All authors approved the final submitted version.

## Conflict of Interest

The authors declare that the research was conducted in the absence of any commercial or financial relationships that could be construed as a potential conflict of interest.

## Publisher's Note

All claims expressed in this article are solely those of the authors and do not necessarily represent those of their affiliated organizations, or those of the publisher, the editors and the reviewers. Any product that may be evaluated in this article, or claim that may be made by its manufacturer, is not guaranteed or endorsed by the publisher.
